# Design of Multimedia English Online Teaching Platform under Wireless Network Communication Technology

**DOI:** 10.1155/2022/1894067

**Published:** 2022-04-23

**Authors:** He Dan

**Affiliations:** Department of College English, Liaoning University of International Business and Economics, Shenyang, China

## Abstract

The traditional online teaching platform has poor compatibility due to the high data delay in practical applications. Therefore, a Multimedia English online teaching platform under wireless network communication technology is designed. Aiming at the actual functional requirements of online teaching, the overall architecture of the Multimedia English online teaching platform is designed. In this architecture, the hardware of the data collector, memory, and main controller is deployed to build the platform. Based on the wireless network communication technology, the software modules are divided into two parts. It is made of a number of functional modules. The design of the platform functional modules is mainly based on the main functions of the administrator submodule, the teacher submodule, and the student submodule. At the same time, the weight of the indicators is determined by combining the analytic hierarchy process and the evaluation domain for the quality evaluation of Multimedia English online teaching is established. The level model completes the platform design. The experimental results show that the test results of the designed platform meet the expected goals and can effectively improve the quality and efficiency of Multimedia English online teaching. The teaching quality is always higher than 95%, and the average teaching efficiency is 96.27%.

## 1. Introduction

In order to improve the stability of the Multimedia English online teaching platform and meet the needs of Multimedia English online teaching in larger colleges, it is really necessary to improve the management mode of resources in the platform [1]. At the same time, how to carry out Multimedia English online teaching in a more vivid form is also the key to improving teaching quality [2, 3]. Wireless network communication technology refers to the long-distance transmission of signals between multiple nodes without transmission through conductors or cables. Wireless network communication can be carried out by using various fixed, mobile, and portable applications, such as two-way radio, mobile phones, personal digital assistants, wireless networks, and radio, which can make students pay more attention to learning situations and minimize the interference of the surrounding environment [4]. The Multimedia English online teaching platform breaks the restrictions of time and space, but it is more dependent on the network environment [5]. Therefore, improving the operation ability of the platform is also the focus of future research [6].

Relevant scholars have carried out research on this; the study in [7] provides a platform for online teaching to adapt to large concurrent visits. The Multimedia online teaching platform is one of the important contents of the Internet plus education platform. Constructing an online teaching platform suitable for large concurrent access is an urgent requirement for the transmission of university information. Compared with the construction of the Multimedia English online teaching platform in colleges and universities under the new situation, there are some new problems. Large concurrent access puts forward new requirements for platform performance, network bandwidth, and teachers' and students' literacy. Based on the new objectives and main problems of educational informatization 2.0, this paper puts forward countermeasures and suggestions from the aspects of new objectives of platform construction, network bandwidth, quality of teachers and students, new platform selection concept, new platform deployment mode, new network unblocked mode, new teaching evaluation method, new quality improvement requirements, etc. The study in [8] puts forward the practice and research of hybrid teaching of sports anatomy courses based on the Multimedia English online teaching platform and demonstrates the superiority and feasibility of the hybrid teaching mode through experimental comparison, mathematical statistics, and literature review. The results show that the students in the experimental group with a mixed teaching mode had better knowledge and understanding of the relevant contents of the experiment than the students in the control group with traditional teaching methods. The mixed teaching mode is especially suitable for the characteristics of students majoring in physical education, and it is worth popularizing and applying in the teaching of sports anatomy.

Although the above research has made some progress, the application under wireless network communication technology is not enough. Therefore, the design of a Multimedia English online teaching platform under wireless network communication technology is proposed. Wireless network communication technology is a communication method for information exchange by using the characteristics that electromagnetic wave signals can propagate in free space. It can be point-to-point communication, point-to-multipoint communication, broadcasting, cellular network, other wireless networks, and WiFi technology. Its application in the Multimedia English online teaching platform had a good effect. Setting the actual functional requirements of online teaching as the goal, the author designs the overall architecture of the Multimedia English online teaching platform, deploys hardware and software modules in this architecture, determines the index weight combined with the analytic hierarchy process, establishes the evaluation-domain level model of Multimedia English online teaching quality evaluation, and completes the design of the Multimedia English Online teaching platform. The results show that the designed platform can meet the expected objectives and improve the quality and efficiency of Multimedia English online teaching.

## 2. Multimedia English Online Teaching Platform Based on Wireless Network Communication Technology

### 2.1. Architecture Design of the Multimedia English Online Teaching Platform

The Multimedia English online teaching platform is based on the open-source platform for architecture and secondary development. In order to standardize the development process and improve the development efficiency, the overall architecture of the Multimedia English online teaching platform is designed with wireless network communication technology to achieve the design goal of the platform [9, 10]. The upper layer does not need to completely rely on the specific implementation details of the lower layer. Changing the structure of the upper layer will not affect the lower layer, making the code more concise, so as to meet the coupling requirements of various modules of the Multimedia English online teaching platform [11].

When the server receives the user's request to access the page, it first loads the global configuration file, initializes the loading core framework, such as data operation, routing, and security, schedules the controller according to the configured route, requests the business logic layer and data layer to load data, and renders the data to the page, thus completing the whole process of request operation and rendering and outputting the data to the page [12, 13]. The overall architecture of the Multimedia English online teaching platform is shown in Figure 1.

As shown in Figure 1, the Multimedia English online teaching platform adopts a hierarchical tree structure design, which can be divided into five modules: user layer, application layer, middle layer, data layer, and basic environment layer for the user [14]. According to the actual functions of these five modules, a Multimedia English online teaching platform is designed.

### 2.2. Platform Hardware Design

Platform hardware refers to the physical equipment that constitutes the computer and is the realistic carrier for the operation of various logic programs. In the Multimedia English online teaching platform [15, 16] designed with wireless network communication technology, the key hardware used includes a data collector, memory, and master controller, which will be analyzed in detail as follows.

#### 2.2.1. Data Collector

The data collector is a programmable logic chip equipped with a crawler program, which can be used to complete the search and collection of user history learning data, including web browsing information, user retrieval keywords, resource download records, exchange and interaction information, and other data that can understand user preferences [17]. The programmable logic chip in this platform is EPM240T100I5N TQFP-100 CPLD. The basic parameters of the chip are shown in Table 1.

According to the basic parameters of the chip in Table 1, it can be seen that the programmable logic chip in the Multimedia English online teaching platform plays an important role and, at the same time, it needs to meet the requirements of low noise and high precision during use.

#### 2.2.2. Storage

Massive English teaching resources and a large amount of user historical behavior data are not enough to be stored only by the storage space carried by the platform itself. Therefore, after the data collector completes a collection task, it is necessary to transfer the collected data to the external memory [18, 19]. The memory in this platform is a disk array with 12 disks, which is equipped with a 4-bit Annapurna Labs Alpine AL-324 ARM@Cortex@-A57 Quad-Core 1.7 GHz processor and 46BDDR4 memory (up to 16 GB) support SATA6Gb/s hard-disk transmission interface to provide faster read and write speed. In addition, two GbE SFP +  and two 2.5Gbe network ports are built in the disk array. Using the disk array can realize the reasonable deployment of the network environment, so as to realize the tasks of copying, saving, repairing, and restoring massive data.

#### 2.2.3. Master Controller

The main controller is the core hardware of the Multimedia English online teaching platform, which is mainly used for the overall operation control of the platform and the execution of various business logic operations [20]. The main controller of this platform is dtb-1022 J1900-embedded industrial computer, and its basic parameters are shown in Table 2.

According to the basic parameters of the embedded industrial computer in Table 2, it can be seen that the power supply, CPU, I/O interface, and other components are centrally installed in a chassis, which has the characteristics of compact structure, small size, and low price and generally adopts an integral structure.

### 2.3. Platform Software Design

In order to further improve the overall function of the Multimedia English online teaching platform [12, 21], the software part of the platform can be divided into three modules: administrator management submodule, teacher management submodule, and student management submodule. The specific module function flow chart is shown in Figure 2.

The specific contents of the platform software design are given as follows.

#### 2.3.1. Administrator Submodule

This module is the manager of the Multimedia English online teaching platform. Its main responsibility is platform maintenance and website management [22, 23], to ensure the stable operation of the platform and the effective development of teachers' teaching interaction. This module is the core part of the whole Multimedia English online teaching platform. The specific functions are described as follows:

1. *Role Division*. When logging into the Multimedia English online teaching platform with the browser for the first time, it is necessary to provide the e-mail and other contact information of new users and realize role matching and authority division for new users according to the information provided by users [24, 25]. For example, if the new user is a teacher, the permissions that the new user can use include applying for adding or deleting courses and uploading teaching resources to the network platform; if the new user is a student, the permissions of the user include online course selection, online testing, and viewing results. At the same time, the administrator has the functions of increasing or decreasing users and managing user-level permissions.
2. *Course Management*. By this function, the administrator can add or delete the function categories in the platform through the actual situation of English teaching. At the same time, the administrator also has the right to move, modify, or import new courses for each function, as well as the right to restore and backup courses [26, 27].
3. *Web Page Setup*. The website administrator can choose to install different skin plug-ins to make the platform layout and appearance design more beautiful.
4. *Other Settings and Information Query*. The website administrator can view the online time, offline time, course selection, and listening and other activities of users on this platform; notices and announcements can be issued on the platform, and multiple information can be accurately managed by using this module. The operation flow chart of the specific administrator submodule is shown in Figure 3.

#### 2.3.2. Teacher Management Submodule

One of the main users of the Multimedia English online teaching platform is teachers. The main responsibility of the design is to provide teachers with various permissions and functions through the platform, which can better complete teaching activities. Using the characteristics of the network platform, we can vividly design the English teaching process and carry out effective interactive activities, so as to achieve the purpose of teaching in a fun manner [28, 29]. The specific functions are described as follows:

1. *Applying for Courses*. After receiving the notice of teaching, teachers can apply for adding new courses through the platform and simply design the new courses. At the same time, they can realize the functions of adding, deleting, modifying, moving, and so on. After the administrator imports the students into the platform in batches, group teaching can be realized according to the situation of the students.
2. *Teaching Design and Organizing Activities*. According to the course content and the characteristics of each course, teachers can upload teaching plans, teaching materials, teaching dynamic videos, teaching courseware, and other resources to the Multimedia English online teaching platform to facilitate the teaching process [30]. Based on the above teaching resources, they can achieve the predesigned teaching purpose, so as to improve the teaching quality and promote students to effectively acquire knowledge.
3. *Online Test Management*. In this function module, teachers can use the topic selection function of the question bank in the module to select the test questions in the question bank by random selection or manual selection to form the test paper. At the same time, teachers can also set the test time, the option of whether to answer again, and the number of answers and have the authority to delete, add, and change the order of the test questions. After the end of the semester teaching course, you can also use the network platform to prepare the final examination paper, in which the objective test questions can be judged by yourself through the platform.
4. *Personal Data Management*. Teachers can view and change personal information and also have the functions of setting up personal microblogs and transmitting personal messages. The specific operation flow of the teacher management submodule is shown in Figure 4.

#### 2.3.3. Student Management Submodule

In the Multimedia English online teaching platform, another main user is students. In order to facilitate students to browse the network platform, functions such as selecting course learning, course's interactive activities, online test answers, and setting up personal data are added to the student management submodule [31, 32]. The specific functions are described as follows:

1. *Course Learning*. After successfully registering new users through the browser, students can view the teaching introduction and courses, as well as all learning courses in the semester.
2. *Teaching Interaction*. In the Multimedia English online teaching platform, according to the scene of teachers' curriculum, students can discuss relevant problems with teachers and other students to realize a series of interactive activities, so as to improve students' learning ability [33].
3. *Online Answers*. In order to understand students' mastery of knowledge, students can conduct online self-evaluation according to the unit test provided by teachers after the unit course. After completing the test, they can also enter the Multimedia English teaching platform to realize the score query function, which can consolidate and review knowledge [34, 35].
4. *Personal Data Management*. Students can change their basic personal information in the Multimedia English online teaching platform and establish a personal learning space according to their interests and hobbies. The specific operation flow of the student management submodule is shown in Figure 5.

To sum up, the overall framework of the Multimedia English online teaching platform is preliminarily designed using wireless network communication technology. On the basis of this framework, each functional module is analyzed and designed in detail. A planning decision-making goal is set as *M*_*b*_, and the expression is as follows:

(1) $$\begin{array}{c} M_{b}=Y_{x}\times Q_{s}. \end{array}$$

Here, *Y*_*x*_ represents the influencing factors and *Q*_*s*_ represents the importance data of *Y*_*x*_ corresponding to the planning objectives. Due to the difference in influence degree of influencing factors on the target *M*_*b*_, it is necessary to compare the influence degree, and all the comparison results can be expressed by *D* matrix:

(2) $$\begin{array}{c} D=\left[\begin{array}{c} d_{11},d_{12},\cdots ,d_{1m}\\ d_{21},d_{22},\cdots ,d_{2m}\\ \;\vdots \vdots \cdots \;\vdots \\ d_{m1},d_{m2},\cdots ,d_{mm} \end{array}\right]. \end{array}$$

Here, *d*_*mm*_ represents the influence degree coefficient in row *m* and column *m*. Assuming that the matrix *D* satisfies the consistency condition, the corresponding solution to the eigenvalue problem is as follows:

(3) $$\begin{array}{c} D^{\prime }=d_{mm}\times R_{u}. \end{array}$$

Here, *R*_*u*_ represents the fuzzy comprehensive evaluation coefficient. The fuzzy comprehensive evaluation method is a mathematical evaluation method. It mainly deals with the fuzzy things in the real world quantitatively through the basic theories and methods of fuzzy mathematics and makes an objective, accurate, and practical Multimedia English online teaching evaluation, so as to effectively solve the problems in the actual teaching process. The basic principle of a fuzzy comprehensive evaluation is as follows: give priority to collecting materials for accurate evaluation of Multimedia English online teaching and determine the main factors and grades of evaluation; then, the weight distribution of the online teaching evaluation index is determined by the above analytic hierarchy process, and the fuzzy mathematical model is established. Assuming that the analytic hierarchy process is used to determine the weight, the evaluation-domain level model is set as follows:

(4) $$\begin{array}{c} A=\left(a_{1},a_{2},\cdots ,a_{n}\right). \end{array}$$

Here, *a*_1_, *a*_2_, and *a*_*n*_ all represent the evaluation grade coefficient. The teaching quality evaluation results of different teachers are obtained through the evaluation-domain level model, and the corresponding improvement measures are given in time combined with the evaluation results to ensure the effective improvement of the quality of the Multimedia English online teaching platform, so as to complete the design of the Multimedia English online teaching platform under the wireless network communication technology.

## 3. Experimental Analysis

In order to verify the feasibility of the designed Multimedia English online teaching platform under wireless network communication technology, the following experiments are designed. Taking the course teaching of a college English major as an example, the teaching content is set as the experimental object. On this basis, combined with the virtual simulation platform, the host used for the test is Microsoft Windows Professional Tomcat7.0 host, using Myeclipsee software as the simulation environment, the database type is SQL SERVER2012 Database 5.3, and the expansion device is Web Server, equipped with FTPServer, Mail Server, and Database Server subplatforms. The platform is controlled using Adobe Dreamweaver CS, PhotoImpactl2, and Acorbat9, the network program language is JSP, and the TCP/IP communication protocol is executed. Other test environments are shown in Table 3.

According to the platform test environment in Table 3, the experiment uses English books in a university library as English teaching resources to test the application performance of the platform. The test process is shown in Figure 6.

Based on the test process of the Multimedia English online teaching platform in Figure 6, the simulation test parameters are set, as shown in Table 4.

In order to verify the practicability of the designed platform, the function and performance of the platform are simulated and tested, respectively. Functional testing is to use test cases to verify the function of the platform. The platform teaching function and platform management function are tested, and the results are shown in Tables 5 and 6.

Through the function tests in Tables 5 and 6, it can be seen that during the operation of the platform data function, the client has relatively completed verification measures. Without going through the server, the client can complete reliable information category calibration, prevent the input of dirty data, ensure the quality of teaching resources of the platform, and quickly save the complete information to the database, All test results are passed, and the test results meet the expected objectives.

In order to further verify the effect of the Multimedia English online teaching platform under wireless network communication technology and compare the teaching quality of three different platforms for testing, 150 students with equivalent academic achievements are selected as the test objects, of which every 50 students are a group, and three different platforms are used to teach the same content, of which the full score of the test score is 100, where 100 ∼ 85 points mean excellent; 84 ∼ 60 points mean qualified; and if the score is below 60, it means unqualified. The comparison results of teaching quality of each teaching platform are given in Figure 7.

By analyzing the experimental data in Figure 7, we can see that the teaching quality of the designed platform is always higher than 95%, while the teaching quality of the platform in reference [7] and the platform in reference [8] is lower than 90%. Our platform uses analytic hierarchy process to evaluate the quality of Multimedia English online teaching, so as to obtain the evaluation results of Multimedia English online teaching in time. Through the evaluation results, the corresponding improvement measures are given in time to ensure the effective improvement of the teaching quality of the designed platform. The student test scores of the designed platform are significantly higher than those of the other two platforms, which shows that the designed platform can obtain more satisfactory teaching results. The following experimental tests compare the teaching efficiency of three different platforms. The specific experimental comparison results are shown in Table 7.

By analyzing the experimental data in Table 7, we can see that the teaching efficiency of each platform is constantly changing with the increase in the number of experiments. The average teaching efficiency of the designed platform is 96.27%, the average teaching efficiency of the platform in reference [7] and the platform in reference [8] are 90.96% and 84.85%, respectively, and the decline trend of literature platform teaching efficiency is very obvious, mainly because the two teaching platforms failed to evaluate the teaching quality in the process of practical application, resulting in the cumbersome whole teaching process; it also proves that it is feasible and effective to add analytic hierarchy process to the designed platform for teaching quality evaluation.

To sum up, the designed Multimedia English online teaching platform under wireless network communication technology has a good effect in practical application and can produce positive results. As a practical technical scheme, it is not something in the abstract thinking stage but something that can be implemented in the industry and has the characteristics of enforceability, reproducibility, and usefulness. Compared with other literature platforms, the teaching quality and teaching effect of the designed platform are better and the performance is improved to a greater extent.

## 4. Conclusions and Prospects

### 4.1. Conclusions

1. During the operation of the data function of the Multimedia English online teaching platform under the designed wireless network communication technology, the client has relatively complete verification measures, which can complete reliable information category calibration and ensure the quality of platform teaching resources. A passing status is presented, and the test results meet the expected goals.
2. The designed platform uses the analytic hierarchy process to evaluate the quality of Multimedia English online teaching and obtains the evaluation results of Multimedia English online teaching in time to ensure that the teaching quality of the designed platform is effectively improved, and more satisfactory teaching results can be obtained.
3. The teaching efficiency of the designed platform is good, and it is effective to add the analytic hierarchy process to the platform to evaluate the teaching quality.

### 4.2. Prospects

Due to the limitation of time and other factors, there are still some deficiencies in the designed platform. The follow-up research will focus on the following aspects:

1. We will expand the scope of research, make teachers give more targeted teaching, and ensure the effective improvement of teaching quality and efficiency
2. In the follow-up, we will comprehensively analyze the learning situation of different students, so that the platform can comprehensively summarize and analyze them and give the corresponding teaching plan in time

## Figures and Tables

**Figure 1:** Overall structure of the Multimedia English online teaching platform.

**Figure 2:** Specific design flow chart of the Multimedia English online teaching module.

**Figure 3:** Operation flow chart of the administrator submodule.

**Figure 4:** Operation flow chart of the teacher management submodule.

**Figure 5:** Operation flow chart of the student management submodule.

**Figure 6:** Test flow chart of the Multimedia English online teaching platform.

**Figure 7:** Comparison results of teaching quality on different platforms.

**Table 1:** Basic parameters of the chip.

Attribute	Parameter
Name	Embedded CPLD
Model	EPM240T100I5N
Encapsulation	100-TQFP
Editable type	Editable in the platform
Delay time	≤4.7 ns
Supply voltage-internal	2.5 V, 3.3 V
Number of logical elements/blocks	240
Number of macrocells	192
I/O count	80
Working temperature	−40°C∼100°C

**Table 2:** Basic parameters of the embedded host controller.

Name	Parameters
CPU	On-board Intel J1900 processor
Memory	One 204 pin DDR3L1600 MHZ SO-DIMM memory socket, maximum 8 G
Display	1 HDM interface, 1 VGA interface
Hard disk	1 SATA interface, 1 msata interface
Network	2 gigabit network ports
Extension	1 half height Mini pcle plug-in
COM	8 COM interfaces
USB	5 USB2 0 interface, 1 usb3 0 interface
GPIO	4-bit DI, 4-bit DO
Audio frequency	Line-in interface, line-out interface
Power support	DC 12V power input
Working temperature	−10°C to 70°C

**Table 3:** Platform test environment.

Name	Parameter
Platform	Windows 10
CPU	Intel Zhiqiang E5-2600
Development tool	Sublime
Deep learning tools	Theano

**Table 4:** Experimental parameters of the platform simulation test.

Name	Parameter	
Average crawl processing time of web crawler nodes	≤2 h	
Enter data batch size	128 Mb	
Training rounds	5 rounds	
Number of different convolution kernels	70	
Convolution kernel type	3 kinds	
Hidden layer size	18 × 2	
Full connection layer	Layer 1 input	128 × L × (18 × 5)
	Layer 1 output	200
	Layer 2 input	200
	Layer 2 output	128 × L × (18 × 5)
	Layer 3 input	200
	Layer 3 output	200

*Note.* L stands for the characteristic scale.

**Table 5:** Platform teaching function test.

Number	Test items	Test method	Result
1	Admin/12345	Is the format correct	Adopt
2	Course view	Whether the course is displayed or not	Adopt
3	Search courses	Can I search	Adopt
4	Job submission	Can I submit normally	Adopt
5	Video playback	Can it play normally	Adopt

**Table 6:** Platform management function test.

Number	Test items	Test method	Result
1	Courseware management	Can you find the required courseware correctly	Adopt
2	User management	Can you effectively query the number of users	Adopt
3	Job management	Can I use keywords to browse jobs	Adopt
4	Online interaction	Can you use this function to complete online topic answers	Adopt

**Table 7:** Comparison results of teaching efficiency of different Multimedia English online teaching platforms.

Number of experiments/frequency	Teaching efficiency of the Multimedia English online teaching platform/%		
	Designed platform	Reference [7] platform	Reference [8] platform
2	99.69	98.63	93.52
4	99.37	96.09	92.03
6	98.44	95.25	90.09
8	97.85	94.59	89.21
10	96.33	93.85	87.63
12	96.12	92.43	85.14
14	95.99	91.52	84.22
16	95.47	89.20	82.30
18	94.58	88.30	80.25
20	94.44	86.72	79.12
22	93.29	83.45	77.41
24	93.65	81.43	77.22
Average value	96.27	90.96	84.85

## Data Availability

The raw data supporting the conclusions of this article will be made available by the author, without undue reservation.

## References

[1] Musa R. J., Ejovi O. M., Oghenerhovweya F. O. (2021). Rethinking the design of English language teaching online using the flipped classroom approach. *Social Science Electronic Publishing*.

[2] Cheung A. (2021). Synchronous online teaching, a blessing or a curse? insights from efl primary students’ interaction during online English lessons. *System*.

[3] Thu N. T. H. (2020). Communication skills and reflection practice in smart English teaching and learning environment: a case study. *International Journal of Emerging Technologies in Learning (iJET)*.

[4] Wilson K. (2020). Balancing the disruptions to the teaching and learning equilibrium-responsive pedagogic approaches to teaching online during the covid-19 pandemic in general chemistry classes at an arabian gulf university. *Journal of Chemical Education*.

[5] Mehrpouyan A., Zakeri E. (2021). Approaches using social media platforms for teaching English literature online. *European Journal of Language and Literature Studies Articles*.

[6] Ho W., Tai K. (2020). Doing expertise multilingually and multimodally in online English teaching videos. *System*.

[7] Xiao X. H., Zhang G. L., Pu H. P. (2021). New thoughts on the construction of college online teaching platform adapting to a large concurrent access. *Creative Education*.

[8] Mirong L (2020). The practice and research of blended teaching of sports anatomy course based on network teaching platform. *Journal of Advances in Education Research*.

[9] Alicia P (2020). Teaching email writing through online teaching platform. *International Journal of Clinical Medicine*.

[10] Vadivel B., Mathuranjali M., Khalil N. R. (2021). Online teaching: insufficient application of technology. *Materials Today Proceedings*.

[11] Munirah R., Refnaldi R. (2020). An evaluation of assessment designed by English language education student taechers during teaching parctice. *Journal of English Language Teaching*.

[12] Al-Habsi T., Al-Busaidi S., Al-Issa A. (2021). Integrating technology in English language teaching through a community of practice in the Sultanate of Oman: implications for policy implementation. *Educational Research for Policy and Practice*.

[13] Yadav M. S., Yadav M. K (2020). Role of the transformational generative grammar and other language learning theories in English language teaching. *SSRN Electronic Journal*.

[14] Ssf H, Ans F (2020). Online teaching during covid-19: how to maintain students motivated in an efl class. *Social Science Electronic Publishing*.

[15] Moteanu N. R. (2021). Teaching and learning techniques for the online environment. how to maintain students’ attention and achieve learning outcomes in a virtual environment using new technology. *International Journal of Innovative Research and Scientific Studies*.

[16] Pineda J. E., Cano L. H. T., Peralta M. A. (2021). An inquiry-based framework for teaching English in synchronous environments. *International Journal of Computer-Assisted Language Learning and Teaching*.

[17] Ennis M. J. (2020). Approaches to English for specific and academic purposes: perspectives on teaching and assessing in tertiary and adult education. *Online Submission*.

[18] Pearson R. J. (2020). Clickers versus plickers: comparing two audience response systems in a smartphone-free teaching environment. *Journal of Chemical Education*.

[19] Öztürk H. A. (2020). My quest for negotiating meaning. Reflections on my dilemmas about practices of English language teaching in public school context in Turkey. *Technium Social Sciences Journal*.

[20] Oeamoum N., Sriwichai C. (2020). Problems and needs in English language teaching from the viewpoints of pre-service English teachers in Thailand. *Asian Journal of Education and Training*.

[21] Bhat M., Palanyswamy H. P., Varsha U. (2021). Development and Validation of an automated Dichotic double word test in Indian English using MATLAB. *International Journal of Pediatric Otorhinolaryngology*.

[22] Lin M., Shi C. H, University H. J (2019). An exploration of objective question assessment of English teaching platform under the background of big data. *Journal of Hubei Open Vocational College*.

[23] Yuan Z. H. (2021). Research and practice of mixed teaching mode of online course—taking the advanced mathematics based on “learning pass + ding talk” as an example. *Creative Education Studies*.

[24] You I., Pau G., Wei W., Fung C. (2020). IEEE access special section editorial: green communications on wireless networks. *IEEE Access*.

[25] Chen H. (2019). The influence of online English writing platform on writing metacognitive strategies and writing performance——a study based on English majors in vocational colleges. *Journal of Shaanxi Xueqian Normal University*.

[26] Chen W., Wang F. (2021). Practical application of wireless communication network multimedia courseware in college basketball teaching. *EURASIP Journal on Wireless Communications and Networking*.

[27] Sartini S. (2020). Kahoot in maritime English teaching: its impact on nautical science cadet’s oral reproduction and vocabulary. *English Language Teaching Educational Journal*.

[28] Desmeules-Trudel F., Joanisse M. F. (2020). Discrimination of four Canadian-French vowels by native Canadian-English listeners. *Journal of the Acoustical Society of America*.

[29] Yan X. X., An X. W., Dai W. B., Sun N. L. (2021). Image segmentation teaching system based on virtual scene fusion. *Computer Simulation*.

[30] Boda P. A., Brown B. (2020). Priming urban learners’ attitudes toward the relevancy of science: a mixed‐methods study testing the importance of context. *Journal of Research in Science Teaching*.

[31] Yastibas A. E. (2020). An anthropocentric approach to evaluate English language teaching course books. *Shanlax International Journal of Education*.

[32] Gan T. (2019). Language regulation in English as a lingua franca: focus on academic spoken discourse. *ELT Journal*.

[33] Tarafdar A., Debnath M., Khatua S., Das R. K (2020). Energy and quality of service-aware virtual machine consolidation in a cloud data center. *The Journal of Supercomputing*.

[34] Gashi L. (2021). Intercultural awareness through English language teaching: the case of kosovo. *Interchange*.

[35] Durand T. G., Visagie L., Booysen M. J. (2019). Evaluation of next-generation low-power communication technology to replace GSM in IoT-applications[J]. *IET Communications*.

